RETRACTED

# Mast Cells in Skin Scarring: A Review of Animal and Human Research

**DOI:** 10.3389/fimmu.2020.552205

**Published:** 2020-09-30

**Authors:** Sara Ud-Din, Traci A. Wilgus, Ardeshir Bayat

**Affiliations:** ^1^Plastic and Reconstructive Surgery Research, Centre for Dermatology Research, NIHR Manchester Biomedical Research Centre, University of Manchester, Manchester, United Kingdom; ^2^Department of Pathology, Wexner Medical Center, The Ohio State University, Columbus, OH, United States; ^3^MRC-SA Wound Healing Unit, Division of Dermatology, University of Cape Town, Cape Town, South Africa

**Keywords:** mast cell, skin scarring, hypertrophic scars, keloid scars, animal/human research, inflammation, cutaneous wound healing, fibrosis

## Abstract

Mast cells (MCs) are an important immune cell type in the skin and play an active role during wound healing. MCs produce mediators that can enhance acute inflammation, stimulate re-epithelialisation as well as angiogenesis, and promote skin scarring. There is also a link between MCs and abnormal pathological cutaneous scarring, with increased numbers of MCs found in hypertrophic scars and keloid disease. However, there has been conflicting data regarding the specific role of MCs in scar formation in both animal and human studies. Whilst animal studies have proved to be valuable in studying the MC phenomenon in wound healing, the appropriate translation of these findings to cutaneous wound healing and scar formation in human subjects remains crucial to elucidate the role of these cells and target treatment effectively. Therefore, this perspective paper will focus on evaluation of the current evidence for the role of MCs in skin scarring in both animals and humans in order to identify common themes and future areas for translational research.

## Introduction

Mast cells (MCs) are immune cells which are present in nearly all tissues, but are prominent in organs that are exposed to the environment such as the skin. They are located close to blood vessels, lymphatic vessels, fibroblasts and nerves (1, 2). MCs arise from the bone marrow and then mature from MC progenitors in the tissues (2). However, the origins of mast cells have long been debated. Early research suggested they are positioned on the common myeloid progenitor or granulocyte/monocyte progenitor branches (3). Whilst later studies imply progenitors originate with basophils and MCs within the granulocyte/monocyte progenitors (4).

MCs are involved in many inflammatory and physiological processes, such as tumor progression, angiogenesis and wound healing (5). They commence their journey from CD34+ /CD117+ stem cells in the bone marrow and then proceed through to differentiation and maturation in the tissue (6) (Figure 1A). In particular, there are high numbers of mature MCs present in the skin (7). Several studies have suggested that fibroblasts may contribute to MC maturation, and cell-cell adhesion as well as fibroblast-derived stem cell factor may induce the MC maturation process (8–10).

RETRACTED

**Figure 1:** **(A)** A diagram displaying that mast cells are immune cells which originate from the stem cells in the bone marrow and they undergo the final stages of differentiation and maturation in their target tissues. They have widespread distribution in nearly all tissues and are often found in close proximity to fibroblasts, blood and lymphatic vessels and nerves. **(B)** Illustrations showing the possible role of mast cells (MC) in various phases of wound healing. (i) In the inflammatory phase, vascular permeability is induced by histamine released from activated mast cells, there is degradation of the extracellular matrix, and recruitment of neutrophils. (ii) In the proliferation phase, collagen synthesis, fibroblast proliferation, and epithelialisation are induced and αSMA is upregulated. (iii) Angiogenesis is stimulated by MC-derived mediators such as tryptase, histamine, and VEGF, and (iv) In the final phases of healing, MC mediators stimulate contraction of αSMA and increased collagen cross-linking.

To date, there has been a number of studies in both animals and humans on the role of MCs in wound healing. When classifying MCs, murine MCs are divided into two main subsets: connective tissue MCs and mucosal MCs (11, 12). Whereas, human MCs demonstrate a diverse population of cells which differ in structure, mediators and surface receptors (13). Two classifications of human MCs have been proposed: MCTC cells which contain tryptase, chymase, and carboxypeptidase and MCT cells that contain predominantly tryptase (14). Whether the different subsets of human MCs are similar to those in mice or other species remains to be fully investigated.

MCs can help initiate inflammation, promote re-epithelialization, and simulate angiogenesis (13, 15–24) (Figure 1B). In the inflammatory phase, vascular permeability is induced by histamine released from activated mast cells, there is degradation of the extracellular matrix and recruitment of neutrophils (17). In the proliferation phase, collagen synthesis is upregulated, and epithelialization is induced (21). MCs produce mediators including epidermal growth factor and keratinocyte growth factor, which stimulate keratinocytes (21). Delayed re-epithelialization has been reported in a study using MC-deficient mice in large excisional wounds (18). Whilst, angiogenesis is stimulated by MC-derived mediators such as tryptase, histamine, and VEGF (23) in the final phases of healing, MC mediators stimulate contraction of αSMA, upregulate fibroblast proliferation, and increase collagen cross-linking (5).

RETRACTED

Moreover, both direct and indirect interactions between MCs and fibroblasts are believed to impact scar formation. Despite our current understanding regarding the role that MCs play and their involvement in many aspects of healing, there is still much that we do not understand about their mechanism of action and how these cells function *in vivo*. Results from animal studies are somewhat variable, and the role of MCs in wound healing may be context-dependent and differ based on the specific mouse strain/wound model used or whether there is underlying diabetes or infection (17–23). In particular, there is a critical lack of human studies investigating the role of MCs in cutaneous skin scarring as studies seem to have focused on the early phases of wound healing (11, 15). Therefore, the aim of this paper is to focus and evaluate the available literature regarding the role of MCs in skin scarring in both animals and human skin in order to identify common themes and future areas for research (Supplementary Table 1).

## Fetal Skin Scarring

It has been reported that cutaneous wounds in the early developmental stages have low levels of inflammation and can heal without a scar and can regenerate hair follicles. Conversely, wounds acquired in the late fetal developmental stages have high levels of inflammation and heal with a fibrotic scar. Indeed, several studies have investigated the role of MCs in changing from scarless healing to fibrotic healing using animal models. This has been studied in a mouse fetal repair model study where embryonic day (E) 15 wounds healed without a scar and E18 wounds healed with a scar (25). Their findings showed that there were fewer MCs which were less mature and there was no degranulation upon wounding in scarless E15 wounds compared to fibrotic wounds produced at E18. Additionally, MC-deficient embryos injured on E18 demonstrated less scarring than embryos with ample MCs at E18, further advocating that MCs may have an important role in the severity of scar formation.

Human models have also been utilized to investigate MCs in fetal vs. adult skin. Walraven et al. (26) studied differences between human fetal and adult skin to identify if there were any immune cells present in human fetal skin at 18–22 weeks. They compared the immune system and its chemokines and their findings demonstrated that the number of Tryptase+-MCs were fewer in fetal compared to adult skin. Other human research corroborated these findings by comparing human fetal skin from 20 to 40 weeks of pregnancy and from deceased humans from 1 day to 85 years of life (27). Tryptase-positive MCs were shown to be rare in the dermis of fetuses or young men. However, as the skin aged, MCs became more commonly identified. There was also a strong correlation between age and number of dermal MCs.

RETRACTED

## Adult Skin Scarring

Some experimental evidence has shown that MCs augment fibroblast activity, which is accountable for collagen deposition and remodeling in the scar formation/remodeling phase of repair (28–30). Some studies have shown changes in collagen in wounds from MC-deficient mice. Less fibrosis was observed at the edges of scald wounds in MC-deficient mice (24). Additionally, other studies have suggested that MCs may affect collagen maturation and remodeling more than collagen production (31, 32). While the majority of animal studies have suggested that MCs promote scar formation, some studies have suggested that MC-deficient mouse strains heal with similar granulation tissue and scar size compared to normal mice (19, 33). Nonetheless, there is no clear objective explanation for the discrepancies in these findings, although this could be attributed to in part on differences between the mouse strains and specific injury models used. Overall, it is difficult to determine how informative the results of these studies are for improving our understanding of the role of MCs function in scar formation and maturation in human skin.

In view of these contradictory findings, our group for the first time, investigated the role of MCs using 24 healthy adult human skin scar samples (biopsies) (*n* = 3 per time point) over 8 weeks of acute cutaneous wound healing and scar formation (Supplementary Figure 1) (66). A range of MC markers were used to perform a number of immunohistochemical stain analyses including tryptase (MCT), chymase (MCC), CKit, and Toluidine blue. Furthermore, we evaluated other immune cell markers (M1/M2 macrophages, langerin, CD8+ cells), angiogenic markers (VEGFA and CD31) and an innervation marker (PGP9.5) to identify if there was a link between MCs and these other key markers (Figure 2A). All MC markers including MCT, MCC, CKit, and Toluidine blue demonstrated that all wounds and scars contained higher levels of MCs compared to uninjured skin (Figure 2B). MCT and MCC demonstrated an increase to week 1 and reduction to week 8. CKit showed higher numbers of MCs in wounds and scars from week 1 to week 8 compared to normal uninjured skin. Toluidine blue displayed the same trend where there were greater numbers of MCs at week 1 with a subsequent reduction to the latter time points. All MC markers demonstrated the greatest increase in number at week 1 compared to uninjured skin (range: 233 to 333%), with a gradual decrease from week 1 to week 8 (range: 87 to 177%). These findings were similar to that of markers of angiogenesis including VEGFA and CD31. VEGF-A showed a sharp increase at the early time points, particularly at week 1 (202% compared to uninjured skin) and a gradual reduction at week 8 with a return to levels similar of those at baseline. CD31 vessel count peaked at week 1 (150%) compared to uninjured skin and decreased over time to week 8. M1 macrophages peaked at week 1 and 2 then reduced thereafter to week 8 and M2 macrophages slowly increased from uninjured skin and showed greatest levels at week 5 where levels reduced thereafter. MCT was associated with innervation marker PGP9.5 and MCs demonstrated close contact with nerves predominantly at later time points. CD8+ cells were greater in wounds and scars compared to uninjured skin with levels increasing at week 5 and reducing to week 8. These findings demonstrated a similar pattern for MC expression in animal studies and will certainly help steer further research in explaining the close association between MCs and innervation as well as angiogenesis.

RETRACTED

**Figure 2:** **(A)** The role of mast cells in skin scarring was evaluated using 24 healthy adult human skin scar samples (sequential temporal biopsies) (*n* = 3 per time point) over 8 weeks of acute cutaneous wound healing (66). A range of mast cell markers were used to perform a number of immunohistochemical stain analyses including tryptase, chymase, CKit, and Toluidine blue. Furthermore, we evaluated a number of other immune cell markers (M1/M2 macrophages, langerin, CD8+ cells), angiogenic markers (VEGFA and CD31) and innervation marker (PGP9.5) to identify if there was a link between mast cells and other key markers. This figure displays a panel of immunohistochemical images demonstrating the trends over 8 weeks. *Key:* • *Mast cell tryptase (MCT):* (MCT: Red fluorophore, DAPI: Blue fluorophore) • *Mast cell chymase (MCC)* • *CKit:* (CKit: Red fluorophore, DAPI: Blue fluorophore) • *Toluidine Blue* • *Protein gene product 9.5 (PGP9.5)*+*MCT:* (PGP9.5: Red fluorophore, MCT: Green fluorophore, DAPI: Blue fluorophore) • *M1 macrophages:* (CD68: Red fluorophore, HLA-DR-DP-DQ: Green fluorophore, DAPI: Blue fluorophore) • *M2 macrophages:* (CD68: Red fluorophore, CD206: Green fluorophore, DAPI: Blue fluorophore) • *CD8*+ *cells*: (CD8+: Red fluorophore, DAPI: Blue fluorophore) • *Langerin* • *Vascular endothelial growth factor-A (VEGF-A)* • *Cluster of differentiation 31 (CD31)* **(B)** A graphical representation of the trends of the aforementioned immunohistochemical markers. All mast cell markers including mast cells tryptase and chymase, CKit and Toluidine blue demonstrated that all wounds and scars contained higher levels of mast cells compared to uninjured skin. All mast cell markers demonstrated the greatest increase in number at week 1 compared to uninjured skin (233%; *P* = 0.009, 333, 285, and 313%, respectively) with a gradual decrease at week 8 (86.7%, 177%, 92%, 100% respectively). These findings were similar to that of angiogenesis markers including VEGFA and CD31, with an increase at week 1 (202%; *P* = 0.007, 150%, respectively) compared to uninjured skin and a reduction to week 8. M1 macrophages linked with this trend with greater increases at the early time points. Mast cell tryptase was co-localized with innervation marker PGP9.5 and demonstrated close contact with nerves predominantly at later time points from week 4, 5, 6, and 8 compared to uninjured skin. All these findings may demonstrate a correlation of mast cells with innervation and angiogenesis. Statistical analysis was performed using a repeated measure ANOVA with a Geisser-Greenhouse's correction combined with a Tukey's multiple comparison test (significance at *p* = 0.01 and *p* < 0.01).

RETRACTED

## Pathological Skin Scarring

### Hypertrophic Scarring

MCs have been suggested to play a role in the development of pathological dermal fibrosis such as in the formation of abnormal skin scars, including hypertrophic scars and keloids. Hypertrophic scars are raised, and highly erythematous although they remain within the confines of the original cutaneous wound site (32, 34). A number of murine models of hypertrophic scars have shown prominent mast cell staining in the scar tissue, with some demonstrating an increased number of MCs present in scar tissue compared to normal skin (35–38). High MC numbers have also been described in large animal models of hypertrophic scarring (39, 40).

Gallant-Behm et al. investigated the use of MC stabilizer ketotifen on wound contraction and skin fibrosis in a pig model (41). They used the Yorkshire pig as it is considered that its injured skin heals similar to that of human skin. In addition, the red Duroc pig was used in this model as this type of animal is able to heal with some characteristics, such as wound/scar contraction, similar to that of human hypertrophic scars. Their results demonstrated that collagen deposition was reduced and wound contraction was lower in red Duroc compared to Yorkshire pigs. In addition, there was no effect on MCs in the Yorkshire pigs normal healing in comparison to the red Duroc pigs which showed significantly higher numbers of tryptase positive MCs in the control group compared to the treatment group. The authors suggested that inhibiting activated MC mediators may aid in the prevention of abnormal skin scarring.

RETRACTED

Human studies in hypertrophic scar patients also corroborated the above findings. It has been reported that MCs are evident in hypertrophic scars. This has been suggested to be due to activation of the TGF-β1/Smad signaling pathway as chymase promotes fibroblasts proliferation and collagen synthesis (42). Others observed an increased number of MCs present in hypertrophic scars compared to normal skin in 38 patients (43). Increased numbers of MCs have been shown in normal cutaneous wound healing. MCs have been thought to peak on days 2 to 3, then gradually return to normal levels over time (43). This reduction in MC numbers in normal healing is different to that of hypertrophic scars, where MC numbers have been found to increase and persist permanently as shown in the above studies.

### Keloid Scarring (Keloid Disease)

Keloids are raised fibroproliferative dermal scars of unknown origin that grow and spread beyond the original site of skin injury and characteristically progressively invade the surrounding healthy cutaneous tissue (44, 45). There is no animal model for keloids as these scars are unique to human skin. Only humans and horses are known to be able to develop excessive granulation tissue following skin injury. The appearance of equine exuberant granulation tissue (EGT) is similar to that of keloids in humans. Both keloids and EGTs have been shown to be influenced by inflammatory cytokines. In a study comparing EGT and keloid, similarities were shown in both EGT and keloid having low numbers of MCs (CD117) present (46). These findings contradict the increased number of MCs in keloid tissue demonstrated in many other research papers in humans which will be discussed in the next paragraph. However, the authors noted a limitation relating to where they took the keloid tissue from and whether it contained involved (central) or uninvolved tissue which could explain why they noted less MCs as the peripheral margins of keloid scars are regarded the most active part of the keloid lesion.

Many human studies have demonstrated an increased number of MCs in keloids (47, 48) with some implicating MC chymase promoting fibroblast proliferation TGF-β1/Smad signaling pathway (49), and immunophenotyping studies showing that degranulated and mature MCs are greatly increased in intralesional and perilesional keloid sites (50). These findings further show that greater numbers of activated MCs implicate inflammation as a key factor in keloid formation. Electron microscopy analysis of keloid dermis showed a close association between fibroblasts and MCs supporting the hypothesis that dysregulation of collagen synthesis can lead to increase in MCs during keloid formation (51). Interestingly, a reduction in MC numbers was observed following application of intralesional cryotherapy to keloid scars which had resulted in improvement of the keloid lesions (52).

RETRACTED

In contradiction to the above findings, one study showed that in keloids the frequency of MCs (using toluidine blue) in the papillary and reticular dermis was significantly lower compared to that of normal skin and lower than in hypertrophic scars and mature scars (53). This was also found in another study which used normal and surgical tissue and hypertrophic and keloid scars and showed that MC chymase was low in all tissue types, MC tryptase displayed low levels in normal tissue and keloids and higher expression in the other tissue types (54). In view of these conflicting results and the low number of human studies, there is a need for further research to evaluate the importance of MCs in abnormal scar types.

## Therapeutic Approaches to Target MCs

A few studies have shown a functional role for MCs by examining the effects of MC stabilizers, tyrosine kinase inhibitors, and other drugs. Mast cell stabilizers prevent degranulation via mechanisms that remain ill-defined (55, 56). Inhibiting MC degranulation using MC stabilizing drugs such as ketotifen has been suggested as a potential therapy for hypertrophic scars in red Duroc pigs (41). Reduced wound contraction and scar formation were reported in pigs treated with ketotifen (41). The effects of another MC stabilizer, disodium cromoglycate (DSCG), which has been shown to inhibit MC degranulation and the release of histamine (57), has been studied in mouse wounds. Application of DSCG demonstrated decreased inflammation, reduced scar width and increased collagen reorganization when evaluated in mice (58). Another study using DSCG in C57BL/6 J mice with implanted meshes showed a reduction in inflammation and fibrosis (59).

Tyrosine kinase inhibitors have also been suggested as an option for treatment of scars (60) although some have been discontinued in patients with impaired wound healing (61). Imatinib, a tyrosine kinase inhibitor that targets cKit signaling, has been shown to reduce mast cell recruitment in skin wounds (59) and to inhibit radiation-induced skin fibrosis in a mouse model (62). Imatinib has also been suggested as a potential therapeutic for keloids (63). Another method has been investigated to reduce fibrosis in tsk (tight skin) mice by using a MC chymase inhibitor which inhibited TGF-β1 activation (64). Most of the available research has been performed in animal models of cutaneous healing, with a distinct lack of human models. Therefore, it is difficult to determine whether these results in animals are translatable to human skin with excessive fibrosis.

RETRACTED

Another class of drugs that appears to target mast cells is epigallocatechin-3-gallate (EGCG) compounds. Our group have previously shown in human skin *ex vivo* models that EGCG has beneficial effects on skin scarring (48, 63). EGCG inhibited keloid scar formation, induced scar shrinkage, decreased proliferation, scar volume, MCs and vessel number (48). In a subsequent *ex vivo* organ culture model study (65), topical application of EGCG reduced the expression of MCs tryptase and chymase in normal skin scars compared with controls. These studies for the first time, demonstrated the role of EGCG in *ex vivo* models of human skin scarring and showed that EGCG had a positive effect on decreasing MCs *ex vivo*. Subsequent to this, our group performed the first reported double-blind randomized controlled trial of topical EGCG in a punch biopsy scar model created in 62 healthy human volunteers. This study showed that MC tryptase and chymase numbers were significantly reduced with EGCG compared to placebo, and this coincided with a statistically significant reduction in scar thickness and an increase in scar elasticity with topical EGCG treatment (66). Catechins have also been shown to inhibit MC-stimulated type I collagen expression in keloid fibroblasts (67). This has been suggested to be due to the dampening activation of the PI3k/Akt/mTOR signaling pathways.

## Proposed Mechanisms

MCs are likely to influence the production of scar tissue through multiple mechanisms, including releasing inflammatory mediators, fibrotic growth factors, and directly interacting with fibroblasts via gap junctions (47, 68–73). It has been suggested that both fibroblasts and MCs must be in contact with each other in order for collagen contraction to occur (72). A rodent derived peritoneal MCs line (RMC-1) and human dermal derived fibroblasts were used to elucidate this phenomenon further and demonstrated that connexin-43 expression has modulatory effects on gap junction communications between MCs and fibroblasts (73). A *Snail*-Tg mouse model of skin fibrosis has been used to investigate the mechanisms regulating mast cell activity (74). This identified a potential role for PAI1 which upregulated ICAM1 expression on dermal fibroblasts, leading to cell-cell adhesion of mast cells. PAI1 regulated MC infiltration to the fibrotic skin indicating that PAI1 is a mediator of fibrosis. These experimental findings may point at a novel way for controlling fibrosis; however, their connection to fibrosis development *in vivo* has not been fully investigated.

RETRACTED

## Discussion

The majority of animal and human studies have shown that MCs promote scar formation. However, the specific role of MCs in scar formation remains unclear in view of contradictory and conflicting data. Both animal and human studies have reported that MC count and activation is less in fetal tissue and therefore wounds heal with little or no scarring, compared with more mature tissues that heal with fibrotic scars. MC degranulation and blocking MC activity have been shown in animal models to decrease the amount of scar tissue production. Nevertheless, there is a lack of specificity with MC stabilizers. In addition, there needs to be more *in vivo* studies in humans to elucidate these effects further.

It will be important to define the mechanisms of how MCs influence fibrosis in order to tailor therapeutic options. Many wound healing studies in mice have relied on MC-deficient mouse models, which all have experimental limitations (75). The most commonly used MC deficient strain to date for wound healing studies is the KitW/W-v strain (24, 31, 33). These mice lack MCs due to a deficiency in KIT, which is a critical receptor for MC growth and survival. However, these mice are also deficient in melanocytes and have reduced numbers of neutrophils and basophils. In general, data from MC deficient mice have to be interpreted with caution and questions remain as to whether findings in these models can be translated to humans. Healing mechanisms also differ between species, such as the Yorkshire pig wound healing resembles normotrophic cutaneous healing in human skin, whilst the red Duroc pig forms contracted scars similar to that of human hypertrophic scars (39). *In vitro* studies have used rodent cell lines and have demonstrated direct interaction between MCs and fibroblasts through gap-junctions, however, their function in the development of scarring in humans *in vivo* remains unknown.

Whilst animal studies have proved to be valuable to uncover the role of MCs in wound healing, the translation of these findings to humans remains ill-defined. It is therefore, crucial to elucidate the exact role and mechanism of mast cells in skin scarring and target appropriate treatment effectively. Further human *in vivo* studies will be needed to determine whether MCs are a feasible target to reduce scar formation and fibrosis and to define the exact mechanisms by which MCs influence scar formation.

## Data Availability Statement

All datasets generated for this study are included in the article/Supplementary Material.

RETRACTED

## Ethics Statement

The studies involving human participants were reviewed and approved by University of Manchester Research Ethics Committee. The patients/participants provided their written informed consent to participate in this study.

## Author Contributions

AB conceived the concept. SU-D drafted the manuscript. AB and TW developed the concept and edited the manuscript.

## Conflict of Interest

The authors declare that the research was conducted in the absence of any commercial or financial relationships that could be construed as a potential conflict of interest.

## Supplementary Material

Supplementary Figure 1 Flowchart demonstrating the methodology of the human skin sample study data. Twenty-four human skin samples were used with *n* = 3 in each time point group. 5 mm skin punch biopsy samples were collected on day 0 and 6mm punch re-biopsy samples were created over the previous scar sites at weekly time points. All samples were placed in formalin, underwent tissue processing and were mounted on glass slides. A number of markers were used for immunohistochemical staining; mast cell tryptase (MCT), mast cell chymase (MCC), Ckit, toluidine blue, pan nerve marker PGP9.5 co-stained with MCT, M1, and M2 macrophages, CD8+ cells, VEGF-A, and CD31 angiogenic markers. All stains were quantified by Definiens® Tissue Studio software. For each batch of microscope slides, whole sections of stained tissue in duplicate were scanned, with exposure settings standardized in order to eliminate variability. Statistical analysis was performed using a repeated measure ANOVA with a Geisser-Greenhouse's correction combined with a Tukey's multiple comparison test (significance at *p* = 0.01 and *p* < 0.01).

Supplementary Table 1 **(a)** A table outlining the role of mast cells in skin scarring in animal research. **(b)** A table outlining the role of mast cells in skin scarring in human research.

## Abbreviations

α-SMA: Alpha-smooth muscle actin
CD: Cluster of differentiation
DSCG: Disodium cromoglycate
EGCG: Epigallocatechin-3-gallate
EGT: Exuberant granulation tissue
ICAM1: Intercellular Adhesion Molecule 1
MC: Mast cells
PAI1: Plasminogen activator inhibitor-1
PGP9.5: Protein gene product 9.5
RMC-1: Rodent mast cell line 1
TGF-β1: Transforming growth factor beta 1
VEGF: Vascular endothelial growth factor
VEGF-A: Vascular endothelial growth factor A.
